RETRACTED

# Comparison of Iliac Bone Transplantation with Bone Transport in the Treatment of Femur Fracture and Bone Defect

**DOI:** 10.1155/2022/5358923

**Published:** 2022-10-03

**Authors:** Wei Huang, Wenfeng Zhu, Wei Lu

**Affiliations:** ^1^Department of Orthopedics and Traumatic Surgery, Nantong Municipal Hospital of Traditional Chinese Medicine, Nantong, Jiangsu, China; ^2^Department of Orthopedics, Shanghai Post and Telecommunication Hospital, Shanghai, China

## Abstract

**Objective:**

To compare the curative effect of iliac bone transplantation with the bone transport in the treatment of femur fracture complicated with a bone defect.

**Methods:**

Patients with femur fractures and defects who were admitted to our hospital from January 1, 2020, to January 31, 2022, and met the inclusion criteria were retrospectively selected and allocated into an iliac bone transplantation group or a bone transport group. The treatment effect and quality of life of the two groups were compared.

**Results:**

A total of 98 patients who met the inclusion standards were enrolled, including 50 cases in the iliac bone transplantation group and 48 cases in the bone transport group. There were no significant differences in IL-6, IL-8, TNF-*α*, visual analog scale (VAS) score, or Japanese Orthopedic Association (JOA) score between the two groups on postsurgical day 1 (*p*=0.051, 0.150, 0.102, 0.564, and 0.826 respectively), but there were significant differences in the above index on postsurgical day 7 (all *p* < 0.01). There were no significant differences in social function, physical function, role function, and cognitive function between the two groups one week after the operation (*p*=0.245, 0.051, 0.102, and 0.067, respectively), but there were significant differences in the above parameters at one month after operation (*p*=0.001, 0.005, 0.005, and 0.001, respectively). The total effective rate of the bone transplantation group was significantly better than that of the iliac bone transplantation group (*p*=0.026). The number of postoperative complications in the bone removal group was significantly fewer than that of the iliac bone graft group (*p*=0.001).

**Conclusion:**

Bone transport is effective in treating femur fractures complicated with bone defects, with fewer postoperative complications.

## 1. Introduction

A femur fracture is a relatively common disease, mainly caused by traffic accidents and falls from height, often accompanied by bone defects. The treatment methods for such patients are complicated; the results are not ideal; and the incidence of disability is high. During surgery, large pieces of sequestrum need to be removed, and local bone defects will also occur during the removal, which has a certain impact on the postoperative recovery of patients [1]. At present, for such patients, autologous iliac bone transplantation is mostly used. Although this method has a certain osteogenic effect, the operation is complicated and the complication rate is high. Bone transplantation is based on the principle of “tension-stress law.” Extracorporeal puncture technology has been used to fix steel nails on the bone at the fracture site and gradually elongate the bone through the force of osteotomy. Both the extension and the compression zone allow callus formation until the bone defect heals [2, 3]. Here, we showed the efficacy of autologous iliac bone transplantation vs. bone transport in the treatment of femur fractures and bone defects.

RETRACTED

## 2. Materials and Methods

### 2.1. Methods

Patients with femur fractures and defects who were admitted to our hospital from January 1, 2020, to January 31, 2022, who met the inclusion criteria were retrospectively selected. All patients in this study gave informed consent, and the patients themselves or their representatives signed the relevant consent forms. The inclusion criteria were as follows: femur fracture with the bone defect; surgical treatment required; and no relevant treatment was performed prior to inclusion in the study. The exclusion criteria were as follows: accompanied by malignant diseases, severe infection, organ failure, malignancy, mental illness, or drug allergy. The study protocol was approved by the institutional ethical committee of our hospital.

Patients in the iliac bone transplantation group received autologous iliac bone transplantation, whereas patients in the bone transport group received surgical bone transport [4]. Patients in both groups were treated with broad-spectrum antibiotics within 2 days of surgery to prevent swelling of the limbs. One week after the operation, the observation group continued to stretch for 5 days on the 8th day, and X-ray examinations were taken to observe the changes in osteotomy distraction. After 5 days of traction, the traction was carried out at a speed of 0.75 mm/day starting from 4 days. An X-ray examination was performed 4 weeks after the operation in the treatment group.

### 2.2. Evaluation of Efficacy

Visual analog scale (VAS) pain scale [5]: 0 is the best, no pain; 1–3 points or less mild pain, tolerable; 4–6 points or the pain is more severe, slightly affecting sleep; and 7–10 points or unbearable severe pain, inability to sleep seriously affects the normal life. The Japanese Orthopedic Association (JOA) score was used to evaluate the treatment efficacy, including subjective symptoms, clinical signs, and daily activities limitation. The total score is 0 to 29 points, and the higher the score, the better the function. The quality of life score (out of 100) was used, including social function, role function, cognitive function, and physical function [6]. The higher the score, the better the quality of life.

RETRACTED

### 2.3. Statistical Methods

The data in this experiment need to be verified by SPSS21.0 software (SPSS, Chicago, IL, USA), in which the count data (*n*, %) were analyzed by *χ*^2^ test, and the continuous data (mean *±* *SD*) were analyzed by *t*-test. *p* < 0.05 (2-tailed) was set as the threshold of statistical significance.

## 3. Results

A total of 98 patients who met the inclusion standards were enrolled. All patients in this study gave informed consent, and the patients themselves or their representatives signed the relevant consent forms. The baseline data of the included subjects are detailed below (Table 1).

### 3.1. Comparison of Inflammatory Factors

On the 1st day after surgery, there was no significant difference in IL-6, IL-8, and TNF-*α* between the study group ((45.85 ± 3.64) (74.41 ± 5.37) and (67.23 ± 6.21)) and the control group ((46.63 ± 2.82), (75.45 ± 5.18) and (67.52 ± 6.31)) (*t* = 2.315, 2.175, 2.452, *p*=0.051, 0.150, 0.102). Seven days after surgery, there were significant differences in IL-6, IL-8, and TNF-*α* between the study group ((22.83 ± 1.35), IL-8 (45.53 ± 3.82) and (42.37 ± 5.36)) and the control group ((28.58 ± 3.26), IL-8 (54.32 ± 4.27) and (55.85 ± 6.24)) (*t* = 11.001, 11.014, 10.310, *p*=0.001, 0.001, 0.000). See Table 2 for details.

### 3.2. Comparison of VAS Score and JOA Score between the Two Groups before and after Surgery

There was no significant difference in the VAS score (7.58 ± 2.13) and JOA score (12.57 ± 0.38) of the study group compared with the control group (7.47 ± 2.25) (12.26 ± 0.50), before surgery (*t* = 1.673, 1.538, *p*=0.564, 0.826). After surgery, the VAS score (4.41 ± 0.56) and JOA score (19.50 ± 0.51) of the study group were significantly different from those of the control group (4.36 ± 0.89) (19.41 ± 0.69) (*t* = 12.274, 8.379, *p*=0.005, 0.000). See Table 3 for details.

### 3.3. Comparison of Quality of Life

One week after operation, there was no significant difference in social function, physical function, role function, and cognitive function between the study group ((63.80 ± 3.62), (64.23 ± 5.51), (67.00 ± 6.02), and (62.97 ± 4.28)) and the control group ((65.61 ± 2.80), (64.35 ± 5.08), (66.53 ± 6.25), and (64.33 ± 3.14)) (*t* = 2.019, 1.631, 1.461, 2.130, *p*=0.245, 0.051, 0.102, and 0.067, respectively). One month after operation, there were significant differences in social function, physical function, role function, and cognitive function between the study group ((82.84 ± 1.15), (84.50 ± 3.80), (83.30 ± 5.38), and (80.61 ± 4.85)) and the control group ((79.13 ± 3.20), (75.44 ± 4.26), (76.82 ± 6.34), and (74.35 ± 3.52)) (*t* = 15.943, 12.005, 13.325, 10.142, *p*=0.001, 0.005, 0.005, and 0.001, respectively). See Table 4 for details.

RETRACTED

### 3.4. Comparison of Treatment Effects

The total effective rate of the bone transplantation group was 93.75% (45/48), which was significantly better than that of the iliac bone transplantation group 78.00% (39/50, *χ*^2^ = 4.961, *p*=0.026, Table 5).

### 3.5. Comparison of Postoperative Complications

Postoperative complications occurred in patients in the bone removal group: delayed fracture union (3 cases), osteoarthritis (6 cases), infection (3 cases), pulmonary embolism (1 case), and the total incidence of complications was 27.08%. Compared with the iliac bone graft group: delayed fracture union (5 cases), osteoarthritis (7 cases), infection (6 cases), pulmonary embolism (3 cases), and the total incidence of complications was 42.00%, there was a significant difference between the two groups (*χ*^2^ = 2.405, *p*=0.121). See Table 6.

## 4. Discussion

Evidence published over the past few decades has led to some consensus on the surgical management of femur fractures. However, in daily clinical practice, the exact choice of the implant is still unclear to the individual surgeon, necessitating the use of an easy-to-use, evidence-based surgical approach that covers all types of femur fractures. Many articles recommend treatment of some aspect of surgery, but only a few authors have published a more or less explicit decision tree algorithm for surgical management of proximal femur fractures [5, 7, 8]. In some Western European countries, national guidelines for many aspects of hip fracture management have evolved over the past decade, including recommendations for surgical options for implants.

In car accidents, femur fracture combined with the bone defect is most common, and in accidents such as falls from height and heavy object crushing, due to the high risk of femur fracture combined with bone defect, the treatment is complicated, the prognosis is poor, and the disability rate is high. Bone displacement is based on bone extension, and 1 mm of bone movement is evidenced every day so that the soft tissue is in a state of tension. Vascular endothelial cells will gradually move to polymorphic mesenchymal cells and to some extent evolve into osteoblasts [9–12].

With the elongation of bone, the callus site changes to a certain extent, and the central fibroblasts gradually differentiate into a parallel structure similar to the bone. Femur fractures and bone defects can be effectively treated by shaping the trabecular plate [13]. Bone grafting can completely eliminate sequestrum and has a traction effect on osteogenesis without artificial bone grafting. Autologous iliac bone transplantation technology builds a three-dimensional structure in the human body through bone tissue, induces bone conduction through osteogenesis, and realizes the fusion of bone junctions. Because the iliac bone contains a large amount of cancellous bone and medullary cavity and because the site where it is located is easy to cut, a good bone connection is formed after transplantation [14, 15]. However, different from the traditional artificial pelvis transplantation, after the autologous iliac bone flap transplantation, the soft tissues such as skin flaps and tendons in the donor and recipient areas must be removed, leading to many incisions, complicated procedures, and long operation times. The amount of bleeding during surgery increases, the incidence of postoperative trauma increases, and the probability of postoperative complications also increase. In the surgical treatment of femur fracture and bone defect, if the wound is large and there are multiple wounds, the blood flow at the fracture will be aggravated, and the surrounding soft tissue will be damaged, easily leading to postoperative infection, and the surrounding tissue will be necrotic or fractured. Healing in this situation is slow or complete recovery is not possible [16, 17]. Because of its simple operation, small trauma, and faster bone repair, bone transplant surgery is used in clinical practice. In this study, the surgical effect of the patients in the bone transport group was better than that in the iliac bone transplantation group, and the recovery indices were also faster than those in the iliac bone transplantation group. The applications of bone transport in other conditions are infections, wound healing problems, or neurological disorders [18–23].

RETRACTED

In conclusion, bone transport is effective in the treatment of femur fracture and bone defects, and the incidence of postoperative complications is low.

## Figures and Tables

**Table 1:** General information of patients.

Characteristics	Iliac bone graft group	Bone transport group	*t/χ* ^*2*^ *value*	*pvalue*
Number of cases	50	48		

Age	36.43 ± 5.43	35.28 ± 6.81	1.812	0.074
Gender			0.397	0.529
Male	26	28		
Female	24	20		

Nationality			2.124	0.000
Han nationality	48	43		
Other	2	5		

Whether they have other bone diseases in the past			0.201	0.654
Yes	0	0		
No	45	45		

Bone defect site			0.544	1.421
Femur condyle	31	27		
Mid femur	19	21		

Smoking			0.521	0.000
Never	34	33		
Have	16	15		

Alcohol drinking			0.142	0.003
Never	21	23		
Have	29	25		

Hypertension/diabetes/cerebrovascular disease			1.244	0.012
None	20	26		
Have	30	22		

**Table 2:** Comparison of inflammatory factors ($\bar{x}\pm s$).

Group	Case	IL-6 (*μ*g/L)		IL-8 (pg/L)		TNF-*α* (ng/L)	
		Day 1 after surgery	Day 7 after surgery	Day 1 after surgery	Day 7 after surgery	Day 1 after surgery	Day 7 after surgery
Iliac bone graft group	50	46.63 ± 2.82	28.58 ± 3.26	75.45 ± 5.18	54.32 ± 4.27	67.52 ± 6.31	55.85 ± 6.24
Bone transport group	48	45.85 ± 3.64	22.83 ± 1.35	74.41 ± 5.37	45.53 ± 3.82	67.23 ± 6.21	42.37 ± 5.36
*T*		2.315	11.001	2.175	11.014	2.452	10.310
*p*		0.051	0.001	0.150	0.001	0.102	0.000

**Table 3:** Comparison of VAS scores and JOA scores between the two groups ($\bar{x}\pm s$).

Group	VAS score		JOA score	
	Before surgery	After surgery	Before surgery	After surgery
Bone transport group (*n* = 48)	7.58 ± 2.13	3.10 ± 0.18	12.57 ± 0.38	23.42 ± 0.36
Iliac bone graft group (*n* = 50)	7.47 ± 2.25	4.41 ± 0.56	12.26 ± 0.50	19.50 ± 0.51
*T*	1.673	12.274	1.538	8.379
*p*	0.564	0.005	0.826	0.000

**Table 4:** Comparison of quality of life between the two groups of patients ($\bar{x}\pm s$).

Group	Social function		Physical function		Role function		Cognitive function	
	1 week after surgery	1 month after surgery	1 week after surgery	1 month after surgery	1 week after surgery	1 month after surgery	1 week after surgery	1 month after surgery
Iliac bone graft group	65.61 ± 2.80	79.13 ± 3.20	64.35 ± 5.08	75.44 ± 4.26	66.53 ± 6.25	76.82 ± 6.34	64.33 ± 3.14	74.35 ± 3.52
Bone transport group	63.80 ± 3.62	82.84 ± 1.15	64.23 ± 5.51	84.50 ± 3.80	67.00 ± 6.02	83.30 ± 5.38	62.97 ± 4.28	80.61 ± 4.85
*T*	2.019	15.943	1.631	12.055	1.461	13.325	2.130	10.142
*p*	0.245	0.001	0.051	0.005	0.102	0.005	0.067	0.001

**Table 5:** Comparison of clinical efficacy between the two groups of patients (cases (%)).

Group	Effective rate	Ineffective rate
Iliac bone graft group (*n* = 50)	39 (78.00)	11 (22.00)
Bone transport group (*n* = 48)	45 (93.75)	3 (6.25)
*χ* ^*2*^	4.961	
*p*	0.026	

**Table 6:** Comparison of postoperative complications between the two groups (cases, %).

Group	Delayed fracture union	Osteoarthritis	Infection	Pulmonary embolism	The total incidence of complications
Iliac bone graft group (*n* = 50)	5 (10.00)	7 (14.00)	6 (12.00)	3 (6.00)	21 (42.00)
Bone transport group (*n* = 48)	3 (6.25)	6 (12.50)	3 (6.25)	1 (2.08)	13 (27.08)
*χ* ^*2*^	—				2.626
*p*	—				0.105

## Data Availability

The data used to support the findings of this study are available from the corresponding author upon request.
